# AT7867 Inhibits the Growth of Colorectal Cancer Stem-Like Cells and Stemness by Regulating the Stem Cell Maintenance Factor Ascl2 and Akt Signaling

**DOI:** 10.1155/2023/4199052

**Published:** 2023-02-14

**Authors:** Yuchen Li, Yun Yuan, Luyao Yang, Hongqing Chen, Xufan Zhang, Tian Wen, Wenhao Liao, Maoyuan Zhao, Ziyi Zhao, Qiongying Hu

**Affiliations:** ^1^Department of Laboratory Medicine, Hospital of Chengdu University of Traditional Chinese Medicine, Chengdu, China; ^2^College of Medical Technology, Chengdu University of Traditional Chinese Medicine, Chengdu, China; ^3^Hospital of Chengdu University of Traditional Chinese Medicine, Chengdu, China; ^4^Traditional Chinese Medicine Regulating Metabolic Diseases Key Laboratory of Sichuan Province, Chengdu, China

## Abstract

Cancer stem cells (CSCs) are the core factors leading to recurrence, insensitivity to radiotherapy and chemotherapy, and immunotherapy resistance in patients with colorectal cancer. AT7867, a potent oral AKT inhibitor, was found to have antitumor activity in colorectal cancer; however, the effect on colorectal cancer stem cells is still unclear. This study was conducted to clarify the molecular mechanism underlying the CSC growth inhibitory effects of AT7867. We cultured colorectal cancer cells (CRCs) in a serum-free medium and enriched colorectal cancer stem cells. Subsequently, the effects of AT7867 on CSCs were analyzed by CCK-8, colony formation, flow cytometry, and immunofluorescence assays. The results indicated that AT7867 induces G2/M phase arrest and cell apoptosis in cancer stem cells. Subsequently, we identified Ascl2 as the main gene affecting the stemness of colorectal cancer in AT7867 by RNA sequencing. The current study showed that Ascl2 is involved in the metastasis, invasion, and proliferation of CRCs. The next experiments demonstrated that overexpression of Ascl2 did affect the therapeutic effect of AT7867 on CRC stemness. Furthermore, compared with other Akt inhibitors, AT7867 could promote the differentiation of colorectal cancer stem cells. Thus, AT7867 might be a potential antitumor drug candidate to treat CRC by targeting CSCs.

## 1. Introduction

Colorectal cancer (CRC) is one of the most common tumors, and it has the second highest mortality rate in the world. With changes in diet and lifestyle, the incidence of colorectal cancer is increasing [1]. At present, the main treatment methods for colorectal cancer include surgical resection, radiotherapy and chemotherapy, and immunotherapy; however, patients often have tumor recurrence and metastasis and poor prognosis [2, 3]. A large number of studies have shown that cancer stem cells (CSCs) are the core factor leading to postoperative recurrence, metastasis, and insensitivity to radiotherapy and chemotherapy in colorectal cancer patients [4].

Cancer stem cells, also known as tumor initiating cells, are a group of tumor cell subsets with self-renewal ability, infinite proliferation ability, and strong antiapoptotic ability [5]. Since Bonnet and Dick first isolated CSCs from human acute myeloid leukemia cells in 1997, CSCs have been found in almost all solid tumors [6, 7], including colorectal cancer [8, 9]. Studies have shown that colorectal cancer stem cells are generated by epigenetic mutations in normal stem cells or progenitor cells. Although the proportion of colorectal cancer stem cells is less than 0.1%, it has been proven that the existence of colorectal cancer stem cells has an impact on the occurrence and development of colorectal cancer, playing an important role in drug resistance, invasion, and metastasis [10, 11]. On the one hand, CSCs are in the G0 dormant phase for a long time, resulting in drug resistance in colorectal cancer. On the other hand, CSCs secrete immunosuppressive cytokines such as TGF-*β*, IL-6, and IL-10 to induce immune escape of tumor cells [12, 13]. Therefore, finding a drug targeting CSC is of great significance for the treatment of colorectal cancer.

At present, it is reported that AT7867 is an effective orally active AKT inhibitor, and it has been confirmed that it has the ability to inhibit tumor cell proliferation and induce tumor cell apoptosis, especially in CRC [14]. Scientists further found that AT7867 promotes apoptosis in colorectal cancer cells by inhibiting SphK1 and blocking AKT-S6K1 activation [15]. In addition, to find an effective small molecule inhibitor for mesenchymal stem cell-like triple-negative breast cancer cells, the You team screened the existing clinical/preclinical protein kinase inhibitors and found that AT7867 was the most effective small molecule inhibitor among them [16]. Although these studies demonstrate that AT7867 has antitumor effects and adjusts stem-like properties, the role and molecular mechanism of AT7867 in CSCs derived from colorectal cancer remain unclear. In this study, we identified the stemness characteristics of CSCs derived from colorectal cancer and the molecular mechanisms underlying AT7867 regulation of CSC proliferation and stemness.

## 2. Materials and Methods

### 2.1. Reagents

For in vitro experiments, AT7867 (APExBIO, China) was dissolved in dimethyl sulfoxide (DMSO) at a stock solution concentration of 10 mmol/L. AT7867 was dissolved in a mixed solution of 10% DMSO, 40% PEG300, 5% Tween80, and 45% saline for in vivo experiments. Miltefosine was purchased from APExBIO (Shanghai, China).

### 2.2. Cell Culture

Colorectal cancer cell lines HCT116 and HT29 were obtained from the Cell Bank of the Chinese Academy of Sciences (Shanghai, China). The cells were cultured in DMEM/F12 (Gibco, USA) medium containing 20 ng/mL epidermal growth factor (EGF) (Invitrogen, USA), 10 ng/mL basic fibroblast growth factor (bFGF) (Invitrogen, USA), and 2% B27 supplement (Gibco, USA), and the medium was changed twice a week. CSCs were passaged every five to seven days.

### 2.3. Limiting Dilution Analysis

We cultured HCT116 and HT29 cells in serum-free medium for 7 days and collected the spheres. Spheres were dissociated into a single-cell suspension. For each passage, the same number of single-cell suspensions was seeded and cultured for addition 7 days in serum-free medium. Then, we made the first-, second-, third-, fourth-, and fifth-generation spheres into single-cell suspensions and inoculated into 6-well plates with 1000 cells per well. Then, they were observed under an inverted microscope. We use the following formula to calculate sphere forming efficiency (SFE): SFE = the number of cells with a diameter greater than 70 *μ*m in each well/the total number of originally seeded cells in each well × 100%.

### 2.4. Western Blot (WB)

After the cells were made into a single-cell suspension with TrypLE (Gibco, USA), loading buffer containing 1% *β*-mercaptoethanol (Solarbio, China) was added to lyse the extracted proteins. Proteins were subsequently loaded into 10% SDS-PAGE and transferred to PVDF membranes. We blocked with TBST containing 3% bovine serum albumin for one hour, followed by incubation with primary antibody overnight at 4°C. Primary antibodies are as follows: Oct4 (Zen-BioScience, China), Nanog (Zen-BioScience, China), CD44 (Abcam, UK), CD133 (Abcam, UK), Ascl2 (CST, USA), Cleaved-PARP (CST, USA), Cleaved-Caspase3 (CST, USA), p21 (Abcam, UK), and *β*-actin (Beyotime, China). Membranes were rinsed, followed by secondary antibody (Beyotime, China) incubation for one hour, and bands were visualized using the ECL detection kit.

### 2.5. Transwell

Cells were made into single-cell suspension, and the cells were resuspended in serum-free DMEM/F12 medium in a Transwell chamber (Corning, USA) at a density of 1 × 10^4^/mL. DMED/F12 containing 10% FBS was added to the bottom of the plate. After 24 h of incubation, Transwell membranes were fixed with 4% paraformaldehyde for 30 min, subsequently stained with crystal violet for 30-45 min, washed with PBS, and allowed to dry. Images of migrated cells were taken under an inverted microscope.

### 2.6. In Vivo Tumorigenesis Analysis

To evaluate the tumorigenicity of CSCs and CRCs. Four- to six-week-old female nude mice were purchased from Tonglihua. Nude mice weighed in the range of 18-22 g. Then, CSCs were made into single-cell suspension, mixed in serum-free DMEM/F12 medium, and implanted subcutaneously on the left and right sides of nude mice (1 × 10^5^). There were 4 nude mice in each group, and tumor growth was observed and recorded twice a week. Mice were sacrificed three weeks later, and tumor tissues were collected for HE staining.

### 2.7. Sphere Formation and Sphere Recovery Assay

CRC-derived CSCs were made into single-cell suspension and seeded in low-adsorption six-well plates at 1 × 10^4^/mL, cultured in serum-free medium, and treated with AT7867. The cells treated with DMSO were used as a control group. After 5 days of incubation in a 37°C incubator, pictures were counted under an inverted microscope. CSCs were treated with different concentrations of AT7867. After 72 hours, cells from each group were collected and digested into single cells. Subsequently, for each group, 1 × 10^4^ viable cells per well were counted and seeded in low-adherent 6-well plates (Corning, USA) in serum-free conditioned medium without AT7867. After 5 days of incubation in a 37°C incubator, pictures were counted under an inverted microscope.

### 2.8. Cell Viability Assay

CSCs were seeded in 96-well plates at 1 × 10^4^ per well, and 200 *μ*L of serum-free medium was added to each well. The cells were treated with 0-25 *μ*M AT7867, and the DMSO-treated cells were used as a control. After incubating at 37°C for 24, 48, and 72 hours, CCK8 reagent (APExBIO, China) was added and the absorbance at 450 nm was measured after incubation for 1 hour. We use the following formula to calculate the cell inhibition ratio: IR = 1 − (absorbance value of treatment group − absorbance of medium/absorbance value of control group − absorbance of medium).

### 2.9. Soft Agar Colony Formation Assay

DMEM/F12 medium containing 0.65% agarose was added to the bottom of the six-well plate. CSCs were seeded in serum-free medium containing 0.35% agarose and placed on top of the bottom layer. Cells were treated with different concentrations of AT7867 for 10 days, and the serum-free conditioned medium without AT7867 was replenished every three days until colonospheres formed. Count was observed under an inverted microscope.

### 2.10. Cell Cycle

After CSCs were treated with different concentrations of AT7867, the cells were separated into single-cell suspensions using TrypLE and collected. Harvested cells were centrifuged at 300 x g for 5 min at room temperature, and cells again washed in PBS and centrifuged at 300 x g for 5 min at room temperature, then fixed with 75% ethanol at 4°C for two hours. Following 3 washes with PBS (centrifuged at 300 x g for 5 min at room temperature), cells were stained in PI staining solution (BD Pharmingen, CA) at 37°C for 30 minutes. We remove the samples for analysis by flow cytometry (Beckman Coulter, USA).

### 2.11. Apoptosis

CSCs were treated with different concentrations of AT7867. After 24 hours, cells from each group were collected and digested into single cells. Cells were washed with PBS and centrifuged at 300 x g for 5 min at room temperature, then mixed in 1 x binding solution and Annexin v and PI (BD Pharmingen, CA) were added. Subsequently, the samples were incubated at room temperature for 15 min and analyzed with a flow cytometer (Beckman Coulter, USA).

### 2.12. Lentiviruses and Transfection

Ascl2 was overexpressed via Ascl2 lentiviral activation particles (GeneCopoeia, Guangzhou, China) per the manufacturer's protocol. Ascl2 encoding gene sequence was cloned by polymerase chain reaction (PCR). Then, Ascl2 lentivirus plasmid was constructed by ligating cloned fragment to lentivirus vector. The Ascl2 lentivirus plasmid and two helper plasmids were transfected into HEK293T cells, using Lipofectamine 2000 (Invitrogen, Carlsbad, CA, USA). Cell supernatant was collected and concentrated after 72 h. The recombinant lentivirus was stored at −80°C, named Ascl2/Lentivirus. HCT116 were infected with Ascl2/Lentivirus. Stable cell models were screened with 5 *μ*g/mL puromycin.

### 2.13. RNA Sequencing

RNA sequencing of control and AT7867-treated HT29 cells (each with 3 biological replicates) was performed using the BGISEQ-500 sequencing system. Gene expression were quantified and normalized using the RSEM tool. Differentially expressed genes (DEGs) between control and AT7867-treated HT29 were screened using the NOISeq method. KEGG pathway enrichment analysis and Gene Ontology analysis of DEGs were conducted.

### 2.14. In Vivo Animal Models and Treatments

Four- to six-week nude mice were purchased from Tonglihua. Nude mice weighed in the range of 18-22 g. All experimental procedures were approved by the Institutional Animal Care and Use Committee of the Institute of Chengdu University of Traditional Chinese Medicine, in compliance with the ARRIVE guidelines and the National Institutes of Health Guide for the Care and Use of Laboratory Animals (NIH Publications No. 8023, revised 1978). The cells were resuspended in DMEM/F12 medium, and CSCs (5 × 10^5^ cells) were seeded subcutaneously on the right side of nude mice. When the average tumor volume reached 60-70 mm^3^, the tumor-bearing mice were randomly divided into three groups of five mice each. These groups included a control group and two AT7867 groups. All mice were treated by intraperitoneal injection every other day for 14 days. Tumor volume was measured every other day using Vernier calipers. Formula: *v* = (*L* × *W*^2^)/2.

### 2.15. Immunofluorescence

Frozen tissue sections were fixed with 4% paraformaldehyde for 40 min, and we permeabilized samples with 1% Triton X-100 for 20 min, which were washed with PBS. Then, the tumor sections were blocked with special blocking buffer (Servicebio, China) for immunostaining at room temperature and incubated overnight at 4°C with primary antibodies: Ascl2 (CST, USA) and Survivin (CST, USA). After letting the slides incubate with the appropriate secondary antibody (CST, USA) for one hour at room temperature, then tissue sections were washed with PBS twice and nuclei were rekindled with DAPI (Servicebio, China). We collect pictures under a fluorescence microscope.

### 2.16. Immunohistochemistry

Cryopreserved tissue sections were fixed with 4% paraformaldehyde and blocked with endogenous peroxidase blocking buffer. The tumor sections were dewaxed using Ventana Ez Prep and endogenous peroxidase quenched with Ventana Universal DAB inhibitor. Slides that were stained for mouse monoclonal primary antibodies were blocked for mouse-on-mouse reactions with AffiniPure Fab Fragment Goat Anti-Mouse IgG (H+L) (Jackson ImmunoResearch Labs Inc., USA) at a concentration of 200 *μ*g/mL diluted in antibody diluent (Beyotime, China) for one hour at room temperature. Sections were incubated with Tunnel or KI67 reaction mixture (Roche, Switzerland) for 1 hour. Sections were rinsed and incubated with Converter-POD for 30 min at 37°C. Sections were stained with DAB substrate and refined with hematoxylin. Counts were observed under a light microscope.

### 2.17. Statistical Analysis

Each experiment was performed at least three times. The software GraphPad Prism software was used for data analysis. Statistical analyses were performed using ANOVA (equal variance) or Welch's ANOVA (unequal variance). A statistically significant difference among groups was defined as *P* < 0.05.

## 3. Result

### 3.1. Sphere Cells Derived from the HCT116 and HT29 Cell Lines Display CSC Characteristics

Sphere cells derived from cancer cells exhibit intensive self-renewal ability and chemoradiotherapy resistance when cultured under specific conditions, such as serum-free medium and low-adsorption substrate [17]. CSCs derived from different colorectal cancer cell lines have different differentiation abilities. Whether differentiation ability affects the enrichment of CSCs, we do not know for the time being. Therefore, we selected the nondifferentiable cell line HCT116 and the moderately differentiable cell line HT29 to enrich CSCs [18]. To enrich stem-like cells, we cultured HCT116 and HT29 cells in DMEM/F12 (containing 2% B27, 10 ng/mL bFGF, and 20 ng/mL EGF) medium for 7 days, and then, we observed spheres of different sizes and floating, shapes (Figure 1(a)). Then, we dissociated the spheres into a single-cell suspension. For each passage, the same number of single-cell suspensions was seeded and cultured for addition 7 days in serum-free medium, and the SFE of each passage increased significantly, potentially due to the increase in stemness of each passage (Figure 1(b)). To evaluate the stemness of the obtained spheres, total protein extracted from spheres at passage 5 was employed to detect stemness markers, including Oct4, Nanog, and CD133. As shown in Figures 1(c) and 1(d), compared to parental cells, spheres presented significantly higher levels of all these proteins. Staining of ALDH, a well-recognized stemness marker of colorectal cancer cells [19], was further evaluated by performing flow cytometry, and it was found that enriched spheres presented a significantly higher ALDH-positive proportion than that of parental cells (Figures 1(e) and 1(f)). The invasive ability of parental cells and sphere cells and tumorigenicity in immunodeficient mice are one of the standard methods for the identification of CSCs [20]. Both HCT116 and HT29 spheres have enhanced invasive capacity compared to parental cells (Figures 1(g) and 1(h)), and sphere cells and parental cells were implanted on the left and right sides of nude mice. On the one hand, as shown in Table 1, it was found that the tumorigenic rate of parental cells was significantly lower than that of sphere cells after injection with the same number of cells. On the other hand, in mice with successful tumor bearing on both the left and right sides, it was found that the sphere cells formed larger tumors than the parental cells (Figure 1(i)). Proving that the sphere cells were more tumorigenic than the parental cells, HE staining (Figure 1(j)) showed that the sphere cells had the same histological features as colorectal cancer. These data suggest that the cultured sphere cells displayed CSC characteristics, so the sphere cells were referred to as CSCs.

### 3.2. Tumor Formation of HCT116 Fifth-Passage Sphere Cells and Parental Cells

#### 3.2.1. AT7867 Inhibits Stemness and the Malignancy of CSCs Derived from HCT116 and HT29 Cells

To determine if AT7867 can inhibit the growth of CSCs, single cells derived from HCT116 and HT29 CSCs were cultured in the presence of 5-30 *μ*M AT7867. We found that AT7867 inhibited the proliferation of CSCs in a concentration-dependent and time-dependent manner (Figures 2(a) and 2(b)). By CCK-8 assay, the dose-response curves showed that the IC50 values of AT7867 in HCT116 CSCs and HT29 CSCs treated for 24 h were 20 *μ*M and 10 *μ*M, respectively. Consistently, HCT116 CSCs were treated at the same concentration (15 *μ*M and 20 *μ*M) and HT29 CSCs were treated at the same concentration (5 *μ*M and 10 *μ*M). Subsequently, we examined the effect of AT7867 on CSC stemness such as sphere formation. CSCs were treated with AT7867, and the results showed that the number and size of CSCs were reduced after five days of treatment. To further determine whether this effect is reversible, we pretreated CSCs for 72 hours, dissociated them into single cells, and cultured them in serum-free medium. After five days, the formation and growth of sphere cells were inhibited (Figures 2(c) and 2(d)). To clarify the mechanism of AT7867 in stemness, we detected stem cell-related markers (OCT4, Nanog, CD44, and CD133) and observed that AT7867 decreased these protein levels in a concentration-dependent manner (Figures 2(a) and 2(f)). Taken together, these data proved that AT7867 not only inhibited CSC proliferation but also CSC stemness.

In addition, the migration and invasion abilities of tumor cells are important indicators to evaluate the malignancy of cancers in vitro. To assess the ability of AT7867 to suppress CSC migration and invasion in vitro, Transwell assays were carried out. AT7867 significantly inhibited invasion ability of CSCs derived from HCT116 and HT29 cells in a dose-dependent manner (Figures 3(a) and 3(c)). Soft agar colony formation assay was used to evaluate the effect of AT7867 on colony formation of CSCs. As the concentration of AT7867 was increased, the CSC clones formed was suppressed in soft agar (Figures 3(b) and 3(d)), showing that AT7867 could inhibit colony formation ability of CSCs. In a nutshell, these results are consistent with the hypothesis that AT7867 prevented tumorigenesis of CSCs by suppressing their invasion and colony-forming abilities.

To further study the effect of AT7867 on CSC proliferation, flow cytometry was used to measure the cycle distribution of CSCs. Following CSCs were treated with different doses of AT7867 for 24 h. It was observed that AT7867 induced CSC G2/M phase arrest (Figures 4(a) and 4(c)). Cell apoptosis is also considered to be the main antiproliferative mechanism of anticancer drugs in tumors. Therefore, we investigated the effect of AT7867 on CSC apoptosis using flow cytometry. AT7867 caused apoptosis in a dose-dependent manner, with apoptosis rates of 21.6% and 27.7% for HCT116 and 17.4% and 24.9% for HT29, respectively (Figures 4(b) and 4(d)). Meanwhile, Western blot analysis was conducted to examine the protein expression level of cell cycle related proteins (p21) and apoptotic proteins (cleaved-caspase 3 and cleaved-PARP). The result showed that the expression of cell cycle inhibitory protein p21 and apoptotic proteins cleaved-caspase 3 and cleaved-PARP levels were increased (Figures 4(e) and 4(f)). Taken together, these results further verified the inhibitory effect of AT7867 on CSC proliferation.

#### 3.2.2. AT7867 Regulates CSC Stemness Expression and Proliferation by Inhibiting the Stem Cell Maintenance Factor Ascl2

To reveal the underlying mechanism by which AT7867 affects CSC stemness, we treated HT29 CSCs with 10 *μ*M AT7867 for RNA sequencing. Human CSC-related pathways were downloaded from the Molecular Signature Database v7.0 (MSigDB), and 456 genes related to CSCs were sorted from the 30 lipid metabolism pathways in Table 2 [21]. The differentially expressed genes (DEGs) were identified based on a false discovery rate threshold of 0.05 and fold change of 2. Here, a total of 456 differentially expressed genes were identified, 8 upregulated genes, and 2 downregulated genes (Figure 5(a)). We analyzed pathways related to CSCs in the Reactome and GO databases. Ascl2 was the most significantly expressed gene in the somatic stem cell population maintenance pathway (Figures 5(b) and 4(c)).

Achaete-scute family bHLH transcription factor 2 (Ascl2) is a member of the basic helix-loop-helix family of transcription factors. Back in the late 1980s, Johnson et al. [22] reported that Ascl2 was mainly expressed in extraembryonic tissues with site specificity. By in situ hybridization and quantitative RT-PCR, it is shown that Ascl2 gene was found to be expressed in the base of the crypt of the large and small intestine and trophectoderm of the placenta, but hardly in other normal tissues. Ascl2 further indicated that its expression was enhanced in benign and malignant neoplastic diseases of the large intestine [23], and its expression alters the hierarchy of stem cells within liver metastases, leading to self-renewal rather than differentiation, thereby affecting tumor clinical behavior [24]. To further clarify the function of the Ascl2 gene in CRC-derived CSCs, compared with parental CRCs, CRC-derived CSCs had higher the protein expression level of Ascl2 and AT7867 could decrease it in a concentration-dependent manner (Figures 6(a) and 6(b)). We next studied the function of Ascl2 in the anticancer effect of AT7867. CSCs efficiently were transfected with Ascl2-overexpressing lentivirus. After 72 hours, the expression of green fluorescence could be observed under a fluorescence microscope. Compared with the control group, the expression of Ascl2 mRNA in the Ascl2 group was significantly increased. Subsequently, HCT116 CSCs were treated at the same concentration (20 *μ*M) and HT29 CSCs were treated at the same concentration (10 *μ*M). As shown in Figures 6(c) and 6(d), Ascl2 overexpression significantly increased the number of sphere cells and reversed the effect of AT7867 on sphere formation. The expression of stemness proteins was detected by WB, and Ascl2 overexpression also reversed the effects of AT7867 on stemness proteins (Figures 6(e) and 6(f)). These data confirmed that the inhibition of cell stemness in AT7867-treated CSCs was attributed to decreased Ascl2 activity.

Since Ascl2 is a key gene in malignancies occurring, we hypothesized that AT7867 can inhibit malignancy occurrence by affecting the activity of Ascl2. We then used flow cytometry to analyze the effect of Ascl2 on HCT116 CSC cell cycle and cell apoptosis. As expected, G2/M phase arrest and CSC apoptosis were induced by AT7867 (20 *μ*M) treatment, and these effects were reversed by Ascl2 overexpression (Figures 7(a) and 7(b)), which showed that Ascl2 affected cell proliferation. We also examined the invasive ability after Ascl2 overexpression. Ascl2 overexpression promoted the invasive ability of CSCs and attenuated the inhibition of the invasive ability of CSCs by AT7867 (Figure 7(c)). These experimental evidences suggested that AT7867 regulated CSC stemness expression and proliferation by inhibiting the stem cell maintenance factor Ascl2.

#### 3.2.3. Anticancer Efficacy of AT7867 on CSCs Derived from CRC Xenografts

To assess the therapeutic effect of AT7867 in vivo, we constructed a subcutaneous colorectal cancer mouse model. CRC-derived CSCs (5 × 10^5^) were inoculated subcutaneously on the right side of each nude mouse. When the tumor size reached 50-70 mm^3^, they were randomly assigned to three groups: control group, 15 mg/kg AT7867 and 25 mg/kg AT7867. The average tumor volume (Figures 8(a) and 8(b)) and tumor weight of mice (Figure 8(c)) in the AT7867-treated group were significantly smaller than those in the control group after 14 days of drug treatment. To investigate the potential antitumor mechanisms of AT7867 in vivo, tumor tissue sections from subcutaneous colorectal cancer mouse model were stained with Ki67, TUNEL, Ascl2, and Survivin. As shown in Figures 8(d) and 8(e), abundant Ki67-, Ascl2-, and Survivin-positive cells and few TUNEL-positive cells were observed in control groups, whereas AT7867 treatment significantly decreased Ki67, Ascl2, and Survivin expressions and increased TUNEL-positive cells. These results implied that AT7867 could inhibit tumor cell proliferation effectively, induce more tumor cell apoptosis, and exert antitumor effect in vivo.

#### 3.2.4. In CRC-Derived CSCs, Survivin Was Activated, and Compared with the Akt Inhibitor Miltefosine, AT7867 Has a Stronger Ability to Inhibit Stemness

The Akt signaling pathway plays a key role in regulating the proliferation, differentiation, and tumorigenic potential of CSCs [25]. Akt activates the antiapoptotic activity of Survivin and makes cancer cells resistant. Studies have shown that lung cancer-derived cancer stem cells have higher expression levels than parental cells [26]. To clarify the expression level of Survivin in CSCs derived from CRCs, we detected the CSC Survivin protein levels. The results indicated that the expression level of Survivin was increased in CSCs compared to parental cells and that AT7867 reduced the expression of Survivin (Figure 9(a)). Studies have shown that both Ascl2 and Survivin are related to the Akt signaling pathway. To further certify that AT7867 has a better effect than other Akt inhibitors in CSCs, we compared AT7867 with miltefosine. Miltefosine, a potent AKT inhibitor, has effects on the self-renewal capacity, cell cycle, and cell apoptosis of colorectal cancer CSCs. We cultured CSCs from low-attachment six-well plates to common six-well plates, and HCT116 cells were treated with DMSO (control), AT7867, and miltefosine. Compared with miltefosine, AT7867 can not only inhibit the formation of sphere cells but also promote CSC differentiation (Figure 9(b)). By WB, we found that AT7867 has a stronger inhibitory effect on the expression of Survivin and Ascl2 (Figures 9(c) and 9(d)). These results indicated that AT7867 would be a promising drug candidate for colorectal cancer therapy in the future.

## 4. Discussion

Colorectal cancer is the third most common cancer type worldwide. Although technological advances in early detection and intervention can improve overall survival in colorectal cancer, due to the presence of CSCs, the prognosis for advanced colorectal cancer patients remains poor [27–29]. Therefore, it is very urgent to find therapeutic drugs for CSCs that are crucial for drug resistance, tumor metastasis, and recurrence. Because colorectal cancer stem cells do not have specific tumor markers and some colorectal cancer cells do not have side population cells [30], the CSCs in HCT116 and HTt29 cell lines learn from the in vitro expansion method of neural stem cells [31]. Colorectal cancer cells were cultured in DMEM/F12 medium containing 2% B27, 10 ng/mL bFGF, and 20 ng/mL EGF, and using a low-adsorption plate, differentiated cells were disrupted in the medium, and undifferentiated cells formed spheres.

Oct4, Nanog, and Ascl2 are the main genes for intestinal stem cells to maintain self-renewal and cell dedifferentiation 32. CD133, CD44, and ALDH are critical surface markers in cancer stem cells [19, 32]. In this study, we found that CSCs derived from CRCs have increased expression levels of stemness genes and tumor stem cell surface markers. In vivo, tumorigenic assays are the standard method to identify CSCs [20], and the tumorigenicity of the fifth-generation sphere cells was significantly higher than that of the parental cells. These data proved that the sphere cells obtained by simulating the expansion of neural stem cells in vitro have the characteristics of CSCs.

The Akt pathway is a signaling pathway that is continuously activated in CSCs and plays an important role in regulating the proliferation, self-renewal, and directed differentiation of colorectal CSCs [33, 34]. Therefore, finding a suitable Akt targeting inhibitor is of great significance in the treatment of CSCs. AT7867, an oral AKT inhibitor, is a particularly potent small molecule inhibitor in mesenchymal stem cell-like breast cancer, but its mechanism of action in CSCs has not been elucidated. In our study, through in vivo and in vitro experiments, we explored the efficacy of AT7867 in the treatment of CSCs, and the results showed that AT7867 inhibited the stemness and malignant tumor behaviors of CSCs in a concentration-dependent manner. Existing studies suggest that Ascl2 has site specificity, which is closely related to the stemness of crypt basal column cells [23, 35]. Decreased Ascl2 gene expression leads to reduced tumorigenicity of colorectal cancer cells and the expression of stemness-related markers [36]. Ascl2 is expected to become a target for colorectal CSC therapy. Our study found that AT7867 can significantly reduce the expression of Ascl2 and Ascl2 overexpression can attenuate the effect of AT7867 on CSCs.

Survivin is the smallest member of the apoptosis-inhibiting family, and it is the most powerful anti-apoptotic protein found thus far. Its antiapoptotic effect is far greater than that of the Bcl-2 family [37]. Overexpression of Survivin can lead to resistance of tumor cells to various chemotherapeutic and proapoptotic drugs [38]. Our team found that colorectal CSCs have higher Survivin expression than colorectal cancer cells by WB, which is one of the reasons for the drug resistance of CSCs. Studies have shown that both Ascl2 and Survivin are related to the Akt signaling pathway [39]. Then, we proved that AT7867 has a strong effect on colorectal CSCs compared with other AKT inhibitors. Miltefosine is a potent AKT inhibitor and has shown potent results in clinical trials in multiple cancers [40]. It is worth noting that miltefosine affects the self-renewal capacity, cell cycle, and cell apoptosis of colorectal CSCs [41]. Therefore, we compared miltefosine with AT7867. We found that AT7867 has a stronger inhibitory effect on Survivin and Ascl2 and can better inhibit the formation of CSCs. In addition, AT7867 can promote the differentiation of CRC-derived CSCs, which miltefosine was not able to do. All the results indicated that AT7867 has great potential for the treatment of colorectal CSCs.

## 5. Conclusions

We found that CSCs were enriched from HCT116 and HT29 cell lines using their ability to form spheres in serum-free conditioned culture. AT7867 suppressed CSCs derived from CRC stemness and proliferation by regulating the stem cell maintenance factor Ascl2 and Akt signaling. Our study demonstrates a potential application for AT7867 in the treatment of CRC via CSC targeting.

## Figures and Tables

**Figure 1:** Sphere cells derived from HCT116 and HT29 cell lines display CSC characteristics. (a) HCT116 and HT29 were cultured in serum-free medium for 14 days to obtain spheres. (b) The SFE of sphere cells from the first to fifth passage. (c, d) The expression of Oct4, Nanog, CD133, and CD44 by performing the Western blot in total protein. (e, f) The ratio of Aldh+ cells was analyzed by flow cytometry assay. (g, h) Transwell assay in fifth-passage sphere cells and the parental cells; the histogram shows the number of migrated cells per field. (i) Representative pictures showing the tumorigenic capacity of 10^4^ fifth-passage CRC sphere cells and 10^4^ parental cells. (j) HE staining of tumor xenografts from the fifth-passage sphere cells. ^∗^*P* < 0.05, ^∗∗^*P* < 0.01, and ^∗∗∗^*P* < 0.001 vs. the parental cells.

**Figure 2:** AT7867 inhibits the growth and stemness of CSCs. (a, b) By being cocultured with AT7867 for 1 to 3 days, cell viability was measured by performing CCK-8 assay. (c, d) Representative morphology after AT7867 treatment (sphere formation assay) or pretreatment (sphere recovery assay); Scale bar 200 *μ*m. (e, f) Oct4, Nanog, CD133, and CD44 protein levels were measured by performing Western blot. ^∗^*P* < 0.05, ^∗∗^*P* < 0.01, and ^∗∗∗^*P* < 0.001 vs. the control.

**Figure 3:** AT7867 inhibits the invasion ability of CSCs. (a–d) CSCs were treated with AT7867 for 24 h. Representative images of colony formation and Transwell. ^∗^*P* < 0.05, ^∗∗^*P* < 0.01, and ^∗∗∗^*P* < 0.001 vs. the control.

**Figure 4:** AT7867 inhibits the proliferation of CSCs (a-d) The cell cycle distribution of CSCs treated with AT7867 was analyzed by flow cytometry and apoptotic cells were detected by Annexin V-FITC and PI double staining, following treatment of CSCs in different doses of AT7867 for 24 h. (e, f) Expression of Cleaved-Caspase 3, Cleaved-PARP and p21 was detected by western blotting in CSCs treated with AT7867. ^∗^*P* < 0.05, ^∗∗^*P* < 0.01, and ^∗∗∗^*P* < 0.001 vs. the control.

**Figure 5:** The differentially expressed genes and signal pathways related to cancer stem cells. (a) Differentially expressed genes between AT7867 10 *μ*M treatment and the control group, with fold change ≥ 2 and *P* value ≤ 0.05. (b) Heatmap colored according to the expression PFKM value, showing all of the differentially expressed genes related to cancer stem cells. (c) Pathway is related to cancer stem cell enrichment analysis of DEGs based on the KEGG database.

**Figure 6:** AT7867 regulates CSC stemness expression by inhibiting Ascl2. (a, b) Western blot detected the parental cells, the fifth spheres, and treatment of the fifth spheres in a different dose of AT7867 expression of Ascl2. CSCs were transfected with Ascl2 vector and then treated with AT7867. (c, d) Representative morphology after AT7867 treatment (sphere formation assay) or pretreatment (sphere recovery assay). (e, f) the expression of Ascl2, Oct4, CD44, and CD133 were detected by western blotting. ^∗^*P* < 0.05, ^∗∗^*P* < 0.01, and ^∗∗∗^*P* < 0.001.

**Figure 7:** AT7867 regulates CSC proliferation by inhibiting Ascl2. (a, b) The cell cycle distribution and cell apoptosis were detected by flow cytometry. (c) Transwell assay was performed to detect invasive assay. ^∗^*P* < 0.05, ^∗∗^*P* < 0.01, and ^∗∗∗^*P* < 0.001.

**Figure 8:** Anticancer efficacy of AT7867 on CSCs derived from CRCs xenografts. (a) Tumors derived from HCT116 CSC-bearing nude mice after 14 days of AT7867 treatment. (b) The growth curves of tumor volume of CSC-bearing mice. (c) Scatter diagrams of tumor weight of H446 CSC-bearing mice. (d, e) Ki67 and TUNEL staining on tumor sections from CSC-bearing mice treated with control, 15 mg/kg, or 25 mg/kg AT7867. (f, g) Immunofluorescent staining of Ascl2 or Survivin on tumor sections from CSC-bearing mice. ^∗^*P* < 0.05, ^∗∗^*P* < 0.01, and ^∗∗∗^*P* < 0.001.

**Figure 9:** In CRC-derived CSCs, Survivin was activated. compared with the Akt inhibitor miltefosine, AT7867 has a stronger ability to inhibit stemness. (a) Western blot detected the parental cells, the fifth spheres, and treatment of the fifth spheres in a different dose of AT7867 expression of Survivin. (b) Representative morphology after AT7867 and miltefosine treatment. (c) The expression of Ascl2 and Survivin was detected by Western blotting. ^∗^*P* < 0.05, ^∗∗^*P* < 0.01, and ^∗∗∗^*P* < 0.001.

**Table 1:** Tumor formation of HCT116 fifth-passage sphere cells and parental cells.

Cell types	10^4^ cells	10^5^ cells
HCT116 5^th^ spheres cells	2/4	4/4
HCT116 parental cells	0/4	1/4

Note: equal numbers (10^4^ and 10^5^) of HCT116 5^th^-passage sphere cells and HCT116 parental cells were implanted simultaneously in the left and right sides of nude mice, respectively. Tumor formation rate was calculated after 4 weeks.

**Table 2:** Pathways related to CSCs in Reactome and GO databases.

Stem cell function-related pathways	Pathway ID	Gene count
GO: somatic stem cell population maintenance	GO:0035019	72
GO: negative regulation of stem cell differentiation	GO:2000737	20
GO: stem cell proliferation	GO:0072089	118
GO: hematopoietic stem cell differentiation	GO:0060218	79
GO: negative regulation of stem cell proliferation	GO:2000647	16
GO: stem cell division	GO:0017145	41
GO: hematopoietic stem cell proliferation	GO:0071425	23
GO: positive regulation of stem cell differentiation	GO:2000738	20
GO: regulation of stem cell population maintenance	GO:2000036	28
GO: neuronal stem cell population maintenance	GO:0097150	22
GO: regulation of stem cell proliferation	GO:0072091	67
GO: somatic stem cell division	GO:0048103	24
GO: stem cell differentiation	GO:0048863	248
GO: positive regulation of stem cell proliferation	GO:2000648	40
GO: regulation of stem cell differentiation	GO:2000736	112
GO: hematopoietic stem cell migration	GO:0035701	6
GO: stem cell fate commitment	GO:0048865	9
GO: mesenchymal stem cell maintenance involved in nephron morphogenesis	GO:0072038	6
GO: mesenchymal stem cell differentiation	GO:0072497	8
GO: mesenchymal stem cell proliferation	GO:0097168	5
GO: asymmetric stem cell division	GO:0098722	10
GO: regulation of hematopoietic stem cell proliferation	GO:1902033	9
GO: positive regulation of hematopoietic stem cell proliferation	GO:1902035	5
GO: negative regulation of stem cell population maintenance	GO:1902455	8
GO: positive regulation of stem cell population maintenance	GO:1902459	8
GO: regulation of somatic stem cell population maintenance	GO:1904672	7
GO: negative regulation of somatic stem cell population maintenance	GO:1904673	5
GO: regulation of stem cell division	GO:2000035	10
GO: regulation of mesenchymal stem cell differentiation	GO:2000739	6
Reactome transcriptional regulation of pluripotent stem cells	R-HSA-452723	31

Note: human CSC-related pathways were downloaded from the Molecular Signature Database v7.0 (MSigDB), and 456 genes related to CSCs were sorted from the 30 lipid metabolism pathways as Liang et al. described previously [21].

## Data Availability

The data presented in this study are available in the paper.

## Abbreviations

CSC: Cancer stem cell
CRC: Colorectal cancer
SFE: Sphere forming efficiency
WB: Western blot
MsigDB: Molecular Signature Database v7.0
DEGs: Differentially expressed genes
Ascl2: Achaete-scute family bHLH transcription factor 2.
